The article "Online Education Satisfaction Assessment Based on Machine Learning Model in Wireless Network Environment" was retracted in 2023. Reasons: signs of a paper mill; suspected computer-generated content; unreliable results or conclusions; concerns about the data.

# Online Education Satisfaction Assessment Based on Machine Learning Model in Wireless Network Environment

**DOI:** 10.1155/2022/7958932

**Published:** 2022-06-29

**Authors:** Jing Qin

**Affiliations:** Criminal Investigation Police University of China, Shenyang, 110854 Liaoning, China

## Abstract

With the development of wireless network technology, the transformation of educational concepts, the upgrading of users' educational needs, and the transformation of lifestyles, online education has made great strides forward. However, due to the rapid growth of online education in my country, many regulatory systems have not kept pace with the development of online education, resulting in low user experience and satisfaction with online education. The establishment of a user satisfaction model is beneficial for attracting attention and thinking about research in the field of online education service quality, assisting enterprises in recognizing the specific impact of various factors in services, accelerating service quality improvement, and assisting in the formulation of industry norms and improving enterprise competitiveness, all of which help students acquire knowledge more easily. In the era of big data, traditional satisfaction evaluation methods have many drawbacks, so more and more machine learning methods are applied to satisfaction evaluation models. This paper takes the research of machine learning algorithm as the core to carry out the research work, uses the cost-sensitive idea to improve the decision tree, considers the cost of different types of classification errors, and uses the random forest principle to integrate the generated decision tree, thereby improving the accuracy of the model. The model has better stability, and the validity of the model is verified by experiments. For a follow-up in-depth investigation of online education satisfaction rating technology, the linked work of this paper has certain reference and reference value.

## 1. Introduction

The use of smartphones and tablet computers has grown in popularity as the mobile Internet has become more popular and network costs for 4G and 5G networks have decreased, and more people are turning to the convenient and fast mobile Internet to access information. “Internet + education” has also emerged, and online education is setting off a profound revolution in learning methods. Online education gives full play to the advantages of wide network dissemination and rapid information update, realizes the sharing of learning resources, and meets the learning needs of learners anytime, anywhere. In recent years, the impact of the pandemic has further promoted the development of online education, and various online education platforms have emerged. However, online education platforms are heating up, and platform competition is escalating, but what follows is that the quality of online education platforms is mixed. Therefore, the analysis of the service quality and user satisfaction of education platforms must be carried out on a daily basis.

How to make online education develop better and faster, benefit more people, and explore issues related to online education satisfaction are of great significance to theoretical basic research, enterprises, and users. The influencing variables of service quality, evaluation methodologies, and evaluation indicators are employed in the online education business on a theoretical foundation. Establishing a sound evaluation index system that adapts to the influencing factors of online education and measures it quantitatively can not only pique everyone's interest and stimulate thought in the field of online education service quality research, but also deepen the subdivision of this subdivision as technical conditions improve. For enterprises, if they recognize the specific influence of various factors in service quality, they can tilt their investment, accelerate the improvement of service quality, improve user satisfaction, enhance the stickiness between users and enterprises, and increase the influence of word-of-mouth communication, which is conducive to formulating the service quality standards of the enterprise or the industry, strengthening the core competitiveness of the enterprise, and improving the industry status of the enterprise. For users, it is possible to gain more knowledge from online learning, and it is more convenient to use. Their explicit and implicit needs can be accurately met. Give full play to the high efficiency and low price of online education, and bring practical convenience to the majority of students. It saves the family's expenses on educational tuition and provides an important supplement to school education. Therefore, online education satisfaction research is a realistic topic.

With the continuous development of scientific computing methods, relevant statistical prediction researchers have turned their attention to the study of machine learning models. In the current era of Internet communication with many data dimensions and huge amounts of data, traditional mathematical statistical models are no longer sufficient to analyze and mine potential mathematical relationships and correlations between independent variables in data. Compared with other traditional statistical models, machine learning models have the following significant advantages: high accuracy, automated calculation, fast calculation speed, and custom features. Common algorithms include decision tree, Bayesian classification algorithm [1], artificial neural network [2], K nearest neighbors [3], and support vector machine [4]. Based on this, this paper establishes a user satisfaction evaluation model based on the decision tree algorithm in machine learning theory and improves the decision tree algorithm.

This research develops a machine learning-based online education satisfaction rating model, presents a decision tree-based mobile Internet satisfaction evaluation model, and enhances the decision tree algorithm. The improved method outperforms the BP neural network algorithm, Bayesian algorithm, and XGBoost algorithm in the experiments.

The paper arrangements are as follows: Section 2 describes the related work.  Section 3 discusses the basic algorithms and principles.  Section 4 examines the satisfaction evaluation algorithm based on decision tree.  Section 5 analyzes the experiments and results.  Section 6 concludes the article.

## 2. Related Work

This section discusses the research on machine learning in the field of customer satisfaction. They analyze the research on user satisfaction of online education.

### 2.1. Research on Machine Learning in the Field of Customer Satisfaction

Liu Yang conducts research on user satisfaction of telecom operators, forms experimental data sets through satisfaction attribute selection and questionnaires, uses random forest algorithm to build prediction models, and uses multi-label classification algorithm to optimize the model [5]. Liu Fan conducts research on user satisfaction in the telecommunications industry and integrates various business processes based on the prediction results of logistic regression to obtain a prediction model of telecommunications user satisfaction [6].

Taking Jingdong Mall as the research object, Fan Miaomiao uses crawler technology to capture a large number of online customer reviews. Through word frequency analysis and topic semantic mining on the content of the reviews, combined with the logistics service satisfaction theory and LDA topic model, the logistics service satisfaction is established.

QIY and LIH have captured the stockholders' evaluations of a company's stock online, quantified the evaluation information using sentiment analysis, and used complex networks to study the conduction characteristics of stockholders' emotions [7]. Schumaker and Chen studied financial news articles through text table features and statistical machine learning and constructed a stock quantitative forecast system based on financial news [8].

Most studies collect data such as consumer behavior records, surveys, and online evaluations and use logistic regression, time series, neural network, and text mining methods to conduct factor analysis and forecast research on customer satisfaction. There is a scarcity of research on consumer satisfaction in online education compared to businesses like telecoms and e-commerce.  Figure 1 show the workflow of machine learning:

### 2.2. Research on User Satisfaction of Online Education

Mei Lick Cheok and Su Luan Wong based on the review of past research on the satisfaction of using information technology system and established a theoretical model of the influencing factors of the satisfaction of online learning in middle school teachers and teaching. Three groups of potential factors affecting secondary school teacher satisfaction were identified. This study proposes a theoretical framework outlining the predictive potential of three key sets of factors for secondary school teachers' online learning satisfaction. It is believed that these factors can be considered when formulating future CPD curriculum and intervention plans and when proposing new curriculum innovations [9, 10].

Eshun and Amofa [11] used an online learning management system to determine the perceived value of multigenerational student groups' educational experiences. They discovered that the curriculum content design of students' online courses, as well as their preference for the classroom environment, resulted in varying levels of student satisfaction and concluded that based on multiple studies. The development of student groups in a contextualized online teaching model can be utilized as a tactic to increase students' learning experience and satisfaction. Kuo et al. [12] tested the student satisfaction model and tested the regression model with a hierarchical linear model, and the results showed that in terms of improving student satisfaction, the improvement of learner interaction with course content was the most promising, while in the course setting, the interaction between learners is negligible. Hsu et al. [13] applied basic psychological needs to online education courses, compared the motivational models of online learning and face-to-face learning, and concluded that whether students' needs are met has an impact on students' learning motivation and learning outcomes. Eom et al. [14] and Harvey et al. [15] used factor analysis and structural equation modeling, respectively, to study the reasons that affect satisfaction and the effect of learning. Eom found that the most important factors affecting the satisfaction of online education platforms and students' learning effects are course design, teacher level and personality, and teacher-student interaction in the classroom; Harvey found that students' satisfaction with online education platforms is not related to the gender of users relationship and found three significant antecedents affecting male and female student satisfaction: word of mouth, facilities, and teachers. Ozyurt [16] collected data using the online education student satisfaction scale and clustered it using the Ward method in the hierarchical clustering method. Graber [17] adopted a quasi-experimental, post hoc comparison research design, using two groups of post hoc tests to compare the effectiveness of brick-and-mortar classrooms and online education in delivering knowledge to students through comprehensive grade point averages, class scores, and student satisfaction survey results. Effectiveness and student satisfaction validate the feasibility of conducting online education, as shown in Figure 2.

Xu Zheng analyzed the characteristics and essence of “Internet +” and regarded “Internet + education” as a kind of integration, which is the deployment and optimization of educational resources once again, which can reduce the entry threshold for users to learn and improve the learning effect. “Internet + education” is O2O under different conditions, with both online supplements and offline foundations. Users of online educational institutions are a special type of users, and their learning and consumption are more passive. Therefore, the teacher's responsibility is not only to simply teach and solve puzzles, but also to supervise and bring about the purpose of students' learning [18].

In the research on user satisfaction evaluation of multimedia courseware resources, Lenny conducted a questionnaire survey on users according to the four influencing factors of multimedia user satisfaction. Its influencing factors are content, interactivity, vividness, and graphic quality [19].

Fernando et al. believed that by surveying learners with distance education experience, they analyzed the influencing factors of distance education user satisfaction: the quality of resource content, the value of content, the availability of resources, and the innovation of resources [20].

The terms “digital natives” and “digital immigrants” were coined by the well-known learning software creator MP Translated (2009) and others to reflect the vast differences in digital technologies between today's individuals and their forefathers. People nowadays want to be a part of new experiences with interactivity, immediacy, virtuality, control, and participation. These all fit perfectly with the characteristics of online education courses [21].

Jon Bergmann and Aaron Sams, according to the educational goal theory of the famous American educational psychologist Benjamin Samuel Bloon, found that although online education methods have adjusted and screened advantageous educational resources, online education can only achieve knowledge and comprehension; there is no guarantee of real outcomes of learning. Jon Bergmann and Aaron Sams then put forward a new educational model theory—Flipped Class. Its core concept is to allow learners to learn actively, participate actively, blended curriculum design and Podcasting classroom [22].

## 3. Basic Algorithms and Principles

Here, it discusses the evaluation method of satisfaction evaluation accuracy. They define the introduction to decision trees.

### 3.1. Evaluation Method of Satisfaction Evaluation Accuracy

The index characteristics of the accuracy, recall, precision, and error rate of the prediction results can usually reflect the good replacement of the model. And these indicator features can be reflected by confusion matrix [23].

Confusion matrix is to analyze the actual value of the sample and the predicted value of the model. If the actual sample is 0, it is a negative example, and if it is 1, it is a positive example. If the predicted class is wrong, it is false, and the prediction is correct, it is real. The final confusion matrix is shown in Table 1.

#### 3.1.1. Accuracy and Error Rate

Accuracy refers to the probability that the model predicts correctly, and its formula is as follows:

(1) $$\begin{array}{c} Accuary=\frac{TP+TN}{C}, \end{array}$$

where *C* is the total number of samples.

Similarly, the error rate refers to the probability that the model predicts incorrectly, and its formula is as follows:

(2) $$\begin{array}{c} \;Error=\frac{FP+FN}{C}. \end{array}$$

#### 3.1.2. Precision and Recall

In practical applications, the accuracy and error rate alone cannot reflect the speed of the model, and customers pay different attention to the positive and negative examples of the target variable. Therefore, we must also consider precision rate.

Precision describes the ratio of the number of samples predicted to be positive and actually positive (TP) to the total number of samples predicted to be positive (*TP* + *FP*)by the model, which is as follows:

(3) $$\begin{array}{c} \;Precision=\frac{TP}{TP+FP}. \end{array}$$

This indicator represents the proportion of samples predicted as positive by the classifier that are actually positive.

Recall describes the ratio of the number of samples that the model predicts to be positive and are actually positive to the total number of samples that are actually positive in the test dataset, which is as follows:

(4) $$\begin{array}{c} Recall=\frac{TP}{TP+TN}. \end{array}$$

This indicator represents the proportion of positive samples that the classifier predicts correctly, accounting for the actual positive samples. Since the positive and negative samples of the data set used in this paper are unbalanced, and the education satisfaction research will pay more attention to those “dissatisfied” user evaluation data, the evaluation criteria of the satisfaction model in this paper are mainly based on recall rate and accuracy rate, as a supplement.

### 3.2. Introduction to Decision Trees

Decision trees use tree structures to model the relationship between sample features and potential outcomes. Among them, each internal node (non-leaf node) represents a test on a feature, each branch represents an output of the test, each leaf node stores a class label, and the vertex of the tree is the root node. As shown in Figure 3, this is a sales decision tree model of a certain product, which predicts whether customers will buy a certain product according to customer characteristics. The rectangles represent the non-leaf nodes of the tree, and the ellipses represent its leaf nodes.

The decision tree processing problem is generally divided into the following two steps:

- First, learn the training set to establish a decision tree classification model
- Use the established decision tree classification model to classify samples of unknown types

#### 3.2.1. Decision Tree Generation

The establishment of a decision tree model is a recursive process that needs to repeatedly decompose the data into smaller subsets, and the process does not stop until the resulting subsets meet a stopping criterion. The root node represents the entire data set. At this time, there is no data decomposition. The decision tree selects a feature to decompose the data set. The first group of decisions is formed by dividing all of the data into separate subsets based on the value of the feature. Continue to decompose the data according to different feature values along each branch until the stopping condition is satisfied. If the node reaches the stop condition and no longer decomposes, the node becomes a leaf node. Each leaf node is a label, and the label is determined according to the category of the instance that is assigned to the node. The result of the decision tree model establishment is to establish a decision tree that can predict and classify unclassified samples, and its establishment process follows the idea of “divide and conquer.” The construction of a decision tree is a recursive process, and the decision tree algorithm returns recursion in three situations:

1. The samples contained in the nodes belong to the same category
2. The current attribute set is an empty set, or all samples in the node have the same value on this attribute
3. The current node does not contain any samples, that is, the sample set is empty

Through the learning of the data set, a tree can be established to classify unknown types of samples. When classifying a sample, first start from the top level of the decision tree, test the attributes of the sample, and judge that the sample should walk down the branch of the decision tree according to the attribute value. Each non-leaf node of the decision tree will test the data attributes until the sample reaches a leaf node of the decision tree and the classification is completed. Then, the type of the sample is the type marked by the leaf node.

#### 3.2.2. Decision-Making Optimal Attributes Selection

The key to the establishment of the decision tree model lies in the selection of the optimal attribute. There are many ways to choose the optimal attribute of the decision tree. The most classic ones are information entropy, information increase, and information gain rate. At the same time, these three concepts are also the cornerstone of ID3 algorithm and C4.5 algorithm. The information gain rate is the splitting index of C4.5. The main function of information entropy is to judge the purity of the sample type in the sample set, assuming the current sample set the proportion of the kth class samples in *D* is *p*_*k*_(*k* = 1, 2, 3, ⋯, |*y*|), then the information entropy of *D* is expressed as

(5) $$\begin{array}{c} Ent\left(D\right)=-\overset{y}{\underset{k=0}{\sum }}p_{k}\log_{2}p_{k}. \end{array}$$

From Formula (5) that when the purity of sample *D* is higher, the value of Ent(D) is smaller, and the minimum value is 0. When the purity of *D* is lower, the value of Ent(D) is larger, and the maximum value is 1.

When using a decision tree algorithm to select optimal attributes, the higher the purity of the target variable, the better. Therefore, the concept of information gain is introduced to measure the effect of splitting according to attributes.

Assuming that the discrete attribute *A* has *v* possible values {*A*_1_, *A*_2_, *A*_3_, ⋯, *A*_*v*_}, if the sample set *D* is divided by the attribute *A*, *v* branch nodes will be generated, of which the *v* branch node contains all the values in the attribute *A* in *D*. The value of the sample *A*_*v*_ is denoted as *D*_*v*_. We can calculate the information entropy of *D*_*v*_according to Equation (5). Considering that the number of samples contained in different branch nodes is different, assign weights to the branch nodes |*D*_*v*_|/|*D*|. *D*indicates the number of samples in the set *D*_*v*_. That is, the branch node with more samples has a greater influence, so the calculation is based on the attribute the information gain obtained by dividing the sample set D by A:

(6) $$\begin{array}{c} Gain\left(D,a\right)=Ent\left(D\right)-\overset{V}{\underset{v=1}{\sum }}\frac{\left|D^{v}\right|}{\left|D\right|}Ent\left(D^{v}\right). \end{array}$$

To a certain extent, the information gain represents the purity improvement brought by classifying the sample set by attributes. That is to say, dividing the samples according to the information gain can increase the proportion of samples of the same type in the samples. As a result, the widely used ID3 method chooses partition attributes based on information gain. Of course, selecting the best attributes for a decision tree is an NP problem, and there are disadvantages to using information gain as the best attribute selection approach for samples: This method tends to choose attributes with more values as split points. To reduce this preference, the C4.5 algorithm refers to the information gain rate as a splitting index to select the optimal splitting attribute. The information gain rate is defined as

(7) $$\begin{array}{c} Gain\_ration\left(D,a\right)=\frac{Gain\left(D,a\right)}{IV\left(a\right)},\\ IV\left(a\right)=-\overset{V}{\underset{v=1}{\sum }}\frac{\left|D^{v}\right|}{\left|D\right|}\log_{2}\frac{\left|D^{v}\right|}{\left|D\right|}. \end{array}$$

According to the different optimal attribute selection criteria, the decision tree algorithm can be divided into three types: ID3, C4.5, and CART [24]. These three decision tree algorithms have become the most classic decision tree algorithms.

## 4. Satisfaction Evaluation Algorithm Based on Decision Tree

This paper mainly uses the decision tree algorithm to establish a satisfaction evaluation model and optimizes it according to the characteristics of the data set so that it has a good classification performance.

### 4.1. C 4.5 Introduction to Algorithms

The C4.5 decision tree algorithm has a good classification effect and visualization effect, so it is widely used. However, due to the imbalance in the number of positive and negative samples in the data set in this paper, it is not possible to directly use the traditional C4.5 decision tree algorithm for modeling. A good classification effect is achieved. The reasons are as follows:

1. The positive and negative samples of the data set used in this paper are extremely unbalanced. The classic C4.5 approach classifies the leaf nodes and prunes the decision tree based on the lowest error rate, biasing the decision tree's prediction result towards the data. There are numerous types. For example, the number of positive samples in a test set is 90, and the number of negative samples is 10. If the model predicts all the samples in the test set as positive samples, the accuracy of the model can also reach 90%. But this obviously does not make any sense. In real life, the cost of misjudging a sample type as another type is different. For example, predicting a cancer patient as a normal person and predicting a normal person as a cancer patient, obviously the former will cause more serious consequences. The cost of misclassification is different, and it is obviously not advisable to use the lowest error rate as the original criterion
2. A vast number of studies reveal that a single machine learning model's classification effect is not perfect, that it is prone to overfitting, and that its classification accuracy is limited regardless of which aspect is improved for a single learner. The model's evaluation accuracy can be improved by combining multiple models. Based on the above points, this paper mainly improves the C4.5 algorithm as follows: (1) Introduce a cost-sensitive mechanism to optimize the algorithm, and (2) use the idea of random forest integrate decision trees

### 4.2. C 4.5 Algorithm Optimization

#### 4.2.1. Cost-Sensitive Decision Tree

The positive and negative samples of the data set used in this paper are unbalanced. The traditional C4.5 decision tree algorithm performs leaf node labeling and model pruning optimization according to the minimum error rate, which cannot meet the requirements of satisfaction evaluation. All this paper introduces a cost-sensitive mechanism. Misclassification of different sorts of samples generates varying costs; hence, it is cost-sensitive. Cost-sensitive decision tree is an extension of decision tree learning, which optimizes the labeling and pruning of leaf nodes based on the minimum misclassification cost, rather than the traditional minimum error rate. In recent years, cost sensitivity has attracted extensive research since it was proposed in 2001 and achieved fruitful research results. Cost sensitivity has become a very effective way to solve the imbalance of sample distribution. This paper uses the cost-sensitive idea to improve the C4.5 decision tree algorithm to achieve a more accurate evaluation of mobile Internet satisfaction. The main ideas are as follows:

1. First, a cost-sensitive mechanism is introduced, and the minimum cost is used as the criterion when marking leaf nodes, rather than the original error rate
2. The construction of the decision tree is ended in advance by setting the minimum number of leaf node samples, avoiding over-fitting caused by over-refinement of the decision tree production process
3. This paper mainly adopts the post-pruning method to prune the decision tree, traverses each node of the decision tree in a bottom-up manner, calculates the misclassification cost of the current node, and then calculates and subtracts a certain branch. The misclassification cost before and after changes. If the pruned decision tree has a lower misclassification cost, it will be pruned, resulting in a smaller decision tree with a lower misclassification cost. Several related concepts are now introduced as follows:

**Definition 1 .**

Error cost matrix: Suppose that there are n kinds of classification marks in the training set T, the *p*_1_, *p*_2_, *p*_3_, ⋯*p*_*n*_ current node is k, then define the cost loss matrix CM as

(8) $$\begin{array}{c} CM=\left[\begin{array}{ccc} 0 & \cdots & P_{1n}\\ \vdots & \ddots & \vdots \\ P_{n1} & \cdots & 0 \end{array}\right]. \end{array}$$

Among them, when *i* is not equal to *j*, it indicates the classification cost generated when *p*_*ij*_ the sample with the *p*_*j*_ actual category is judged to be a category *p*_*i*_. When *i* = *j*, it indicates that the current node is correctly classified, and there is no misclassification cost, so it is 0.In leaf node labeling algorithm, the decision tree algorithm will return recursion in three cases:

1. The samples contained in the nodes belong to the same category
2. The current attribute set is an empty set, or all samples in the node have the same value on this attribute
3. The current node does not contain any samples, that is, the sample set is empty

**Definition 2 .**

Node misclassification cost: Assuming that the training set is *T*, there are *m* types in a node of the generated decision tree, and their category flags are, respectively, *p*_1_, *p*_2_, *p*_3_, *p*_4_, ⋯, *p*_*m*_, and the number of samples in each category is *n*_1_, *n*_2_, *n*_3_, ⋯, *n*_*m*_. Assuming that the type of decision tree marked for the current node is *p*_*i*_, the misclassification cost (CL) of its node is defined as

(9) $$\begin{array}{c} CL=\overset{m}{\underset{k=1}{\sum }}n_{k}*p_{ki}. \end{array}$$

In order to prevent overfitting caused by too many branches of the decision tree, this paper adds a recursive return condition, that is, to set the minimum number of leaf node samples min_Num, when the sample contained in the current node is less than min_Num, the recursion ends, and the node is marked as a leaf node. The labeled class is the class with the least classification cost.

In decision tree pruning, the traditional post-pruning method is to first generate a complete tree from the training set and then judge whether to prune according to the lowest classification error rate. If the error rate after pruning is lower than the error rate before pruning, this subtree is replaced with a leaf node, and the type of the node is marked as the type with the most samples. Pruning is not done if the mistake rate after pruning is higher than the error rate before pruning. The typical pruning method ignores the various costs associated with various types of misclassification. This paper improves the traditional pruning algorithm by considering the cost of various types of misclassification.

The specific pruning process is as follows: starting from the leaf node of the decision tree, each inner node of each layer is judged from bottom to top.

  Step 1: Calculate the misclassification cost of each subtree node that may be pruned according to Formula (1)
  Step 2: Calculate the misclassification cost of the subtree if it is not pruned according to Formula (2)
  Step 3: Compare the misclassification cost of the subtree with the misclassification cost after the subtree is pruned and marked as a leaf node. If the former is greater than the latter, the subtree is turned into a leaf node, and the node is marked according to the minimum misclassification cost
  Step 4: Repeat the above process until continuing pruning will increase the misclassification cost

The decision tree pruning can not only generate a decision tree with smaller scale and better generalization performance, but also can increase the number of classification of minority class samples by introducing the idea of cost sensitivity.

#### 4.2.2. Ensemble Method Based on Random Forest

Many studies have proven that a single learner can no longer match people's categorization criteria, necessitating the use of numerous classifiers to create a high-performance combination model, or ensemble learning approach.  Figure 4 depicts the overall architecture of ensemble learning. The integration method in this paper adopts the idea of random forest to integrate the optimized decision tree generated by training.

Random forest is a variant [25], which mainly introduces random attribute selection on the basis of bagging ensemble. The basic idea of random forest is as follows: First, use the bootstrap sampling method to extract k sample sets from the original data set, and then establish k decision tree models for these k sample sets, respectively. Because random forests introduce random attribute selection, for each node of each decision tree, first randomly select a subset of the attributes from the node's attribute set as an attribute subset, and then partition the subset into optimal attributes. In the final prediction, the prediction results of the k decision trees are integrated by voting. The main idea of random forest is shown in Figure 5.

The data set used in this paper has the problem of imbalance of positive and negative samples. Although a cost -sensitive mechanism is introduced in Section 4.2.2, due to the large gap between positive and negative sample data, the corresponding value in the corresponding cost matrix is misclassified. It will also be very vast, resulting in a high error rate and a lot of unpredictability, even though the cost-sensitive decision tree can classify rare class samples well. Furthermore, the data set in this paper is very large. If the model is trained on the original data set, the time efficiency will be very low. Therefore, before generating the cost-sensitive decision tree, this paper uses the sampling method to reduce the positive and negative ratio of the training samples. The specific implementation is as follows: random forest for random sampling of datasets, the data which are first divided into large class datasets and rare class datasets by type .Then, random sampling is performed on the large class dataset and rare class dataset respectively. Then, the randomly sampled sets are combined into a decision tree training set, as shown in Figure 6. The steps of the random forest ensemble method in this paper are as follows:

  Step 1: Input the sample set D, and divide the sample set D into large class sample sets *D*_1_ and rare class sample sets *D*_2_
  Step 2: Perform random sampling with replacement in *D*_1_′ proportion to the large sample set to generate a new sample set. Perform random sampling with replacement *P*_1_ in proportion to the rare sample set to *P*_2_ generate a new sample set*D*_2_′
  Step 3: Combine the sample set *D*_1_′ and *D*_2_′, and combine the decision tree training set
  Step 4: If the sample data contains *n* attribute values, then the decision tree randomly selects *m* attributes (*m* < *n*) during node splitting and selects the optimal attribute for division on this *m* attributes
  Step 5: Repeat Steps 2–4 to generate *k* decision trees

  Step 6: Summarize the classification results of the *k* decision trees. The way of summarizing is to use the method of “majority voting” to determine the final classification result

## 5. Experiments and Results

This section examines the integrated learning. They analyze the comparison of other algorithms.

### 5.1. Integrated Learning

In this paper, the ensemble learning adopts the idea of random forest to integrate the decision tree model. The steps are when randomly sampling the data set, first divide the data into large-class data sets and rare-class data sets by type, and then separate the large-class samples. Sets and rare class samples are sampled, and finally the sampled data sets are combined for decision tree training.

In the experiment, the ratio of positive and negative samples in the training set of a decision tree is 20 : 1, and the number of experiments is 10 times. The performance comparison of each algorithm is shown in Table 2.  Figure 7 shows the recall comparison between algorithms, and Figure 8 shows the accuracy comparison between algorithms.

From Table 2 that the cost-sensitive decision tree can greatly improve the recall rate of the model, but the range of its accuracy and recall rate fluctuates greatly. After the decision tree model integrates the classification results based on the random forest method, although the recall rate cannot be significantly improved, the accuracy and recall rate fluctuate less. Therefore, using the random forest method to integrate the decision tree model can not only improve the accuracy of the model, but also increase the stability of the model.

### 5.2. Comparison of Other Algorithms

Finally, in order to verify the performance of the algorithm in this paper, compared with other mainstream classification learners, other algorithms are used: BP neural network algorithm, Elman neural network algorithm, mlp multilayer perceptron, naive Bayes, XGBoost algorithm.

The algorithm optimized in this study does not have the best accuracy or recall when compared to other algorithms, but it does have the highest F1 source, as seen in Figure 9. That is to say, this paper introduces cost-sensitive ideas to improve the algorithm, which can more accurately find customers who evaluate the mobile Internet as “dissatisfied”. The model has better classification performance.

## 6. Conclusion

The traditional education sector has been greatly influenced by the online education industry. With the rapid advancement of Internet and mobile terminal technologies, the online education market has seen the introduction of more and better course items. The cost of instruction is lower, delivery is more efficient, and the dispersion is wider. However, there is still a lot of room for improvement in customer satisfaction in the current online education industry, and the combination of education and the Internet is still being explored. To this end, this paper establishes an online education satisfaction evaluation model based on machine learning algorithms, proposes a mobile Internet satisfaction evaluation model based on decision tree, and improves the decision tree algorithm. The experimental results show that the optimized algorithm is better than BP neural network algorithm, Bayesian algorithm, and XGBoost algorithm. This model offers a lot of practical value, as well as some reference value and relevance for improving customer satisfaction in domestic online education enterprises.

## Figures and Tables

**Figure 1:** Machine learning workflow.

**Figure 2:** Online education user satisfaction evaluation index model.

**Figure 3:** Decision tree model.

**Figure 4:** Ensemble learning model.

**Figure 5:** Random forest algorithm model.

**Figure 6:** Sampling.

**Figure 7:** Recall comparison.

**Figure 8:** Accuracy comparison.

**Figure 9:** Compare with other algorithms.

**Table 1:** Con fusion matrix.

		True class	
		0	1
Predicted class	0	TN	FN
	1	FP	TP

**Table 2:** Algorithm performance comparison.

	C4.5		Cost-sensitive decision tree		Random forest	
	Accuracy	Recall	Accuracy	Recall	Accuracy	Recall
1	0.9637	0.3118	0.8110	0.6058	0.9011	0.7158
2	0.9642	0.3574	0.7522	0.7623	0.8322	0.7521
3	0.9634	0.3234	0.7942	0.7221	0.8042	0.7408
4	0.9637	0.3834	0.7866	0.7208	0.7966	0.7565
5	0.9642	0.3534	0.8366	0.6765	0.8409	0.7508
6	0.9634	0.3334	0.8166	0.7008	0.8242	0.7367
7	0.9637	0.3634	0.7966	0.6901	0.8342	0.7408
8	0.9642	0.3834	0.7966	0.7208	0.8366	0.7208
9	0.9634	0.3334	0.8266	0.6208	0.8766	0.7308
10	0.9615	0.3234	0.8166	0.7108	0.8205	0.7367
Average value	0.9635	0.3466	0.8225	0.6931	0.8205	0.7367
Standard deviation	0.000789	0.02406	0.04314	0.04547	0.01653	0.0134

## Data Availability

The data sets used during the current study are available from the corresponding author on reasonable request.

## References

[1] Friedman N., Geiger D., Goldszmidt M. (1997). Bayesian network classifiers. *Machine Learning*.

[2] Pearlmutter A. (1989). Learning state space trajectories in recurrent neural networks. *Neural Computation*.

[3] Cover T., Hart P. (1967). Nearest neighbor pattern classification. *IEEE Transactions on Information Theory*.

[4] Joachims T., Finley T., Yu J. (2009). Cutting-plane training of structural SVMs. *Machine Learning*.

[5] Polce M., Kunze N., Fu C. (2021). Development of supervised machine learning algorithms for prediction of satisfaction at 2 years following total shoulder arthroplasty. *Journal of Shoulder and Elbow Surgery*.

[6] Farooq H., Deckard E. R., Ziemba-Davis M., Madsen A., Meneghini R. M. (2020). Predictors of patient satisfaction following primary total knee arthroplasty: results from a traditional statistical model and a machine learning algorithm. *The Journal of Arthroplasty*.

[7] Qi Y., Li H., Liu N., Hao X., Guan Q. (2018). Transmission characteristics of investor sentiment for energy stocks from the perspective of a complex network. *Journal of Statistical Mechanics: Theory and Experiment*.

[8] Schumaker P., Chen H. (2009). A quantitative stock prediction system based on financial news. *Information Processing & Management*.

[9] Cheok L., Wong L. (2015). Predictors of e-learning satisfaction in teaching and learning for school teachers: a literature review. *International Journal of Instruction*.

[10] Matsatsinis F., Grigoroudis E., Delias P. (2003). User satisfaction and e-learning systems: towards a multi-criteria evaluation methodology. *Operational Research*.

[11] Yawson E., Yamoah A. (2020). Understanding satisfaction essentials of E-learning in higher education: a multi-generational cohort perspective. *Heliyon*.

[12] Kuo C., Walker E., Schroder E., Belland B. R. (2014). Interaction, Internet self-efficacy, and self-regulated learning as predictors of student satisfaction in online education courses. *The Internet and Higher Education*.

[13] Wang C., Hsu K., Bonem M. (2019). Need satisfaction and need dissatisfaction: a comparative study of online and face-to-face learning contexts. *Computers in Human Behavior*.

[14] Eom B., Wen J., Ashill N. (2006). The determinants of students’ perceived learning outcomes and satisfaction in university online education: an empirical investigation. *Decision Sciences Journal of Innovative Education*.

[15] Harvey L., Parahoo S., Santally M. (2017). Should gender differences be considered when assessing student satisfaction in the online learning environment for millennials. *Higher Education Quarterly*.

[16] Ozyurt H. (2014). Satisfaction clustering analysis of distance education computer programming students: a sample of Karadeniz Technical University. *Turkish Online Journal of Distance Education*.

[17] Graber J. (2019). Comparison of mental health nursing student academic achievement and satisfaction: classroom versus online education in teaching therapeutic crisis management techniques. *Issues in Mental Health Nursing*.

[18] Sun D., Li S., Xu X. (2020). Analysis of reform and development strategies of China’s internet innovation and entrepreneurship education. *Entrepreneurship Education*.

[19] Khedif B., Engkamat A., Jack S. (2014). The evaluation of users’ satisfaction towards the multimedia elements in a courseware. *Procedia-Social and Behavioral Sciences*.

[20] de Melo Pereira F. A., Ramos A. S., Gouvêa M. A., da Costa M. F. (2015). Satisfaction and continuous use intention of e-learning service in Brazilian public organizations. *Computers in Human Behavior*.

[21] Prensky H. (2009). Sapiens digital: from digital immigrants and digital natives to digital wisdom. *Innovate: journal of online education*.

[22] Sams A., Bergmann J. (2013). Flip your students’ learning. *Educational Leadership*.

[23] Yinghui K., Meili J. (2012). Research on classification method based on confusion matrix and integrated learning. *Computer Engineering & Science*.

[24] Loh Y. (2011). Classification and regression trees. *Wiley interdisciplinary reviews: data mining and knowledge discovery*.

[25] Breiman L. (2001). Random forests. *Machine Learning*.

